# Extracellular Vesicles Carry lncRNA SNHG16 to Promote Metastasis of Breast Cancer Cells *via* the miR-892b/PPAPDC1A Axis

This article has been retracted.

**DOI:** 10.3389/fcell.2021.628573

**Published:** 2021-06-25

**Authors:** Wenfei Xia, Yun Liu, Teng Cheng, Tao Xu, Menglu Dong, Xiaopeng Hu

**Affiliations:** ^1^Department of Breast and Thyroid Surgery, Division of General Surgery, Tongji Hospital, Tongji Medical College, Huazhong University of Science and Technology, Wuhan, China; ^2^Department of ENT, Tongji Hospital, Tongji Medical College, Huazhong University of Science and Technology, Wuhan, China

**Keywords:** extracellular vesicle, lncRNA SNHG16, breast cancer, competing endogenous RNA, miR-892b, PPAPDC1A, bioinformatics analysis

## Abstract

Breast cancer (BC) represents the most commonly diagnosed malignancy among women. Long non-coding RNAs (lncRNAs) can be transferred by extracellular vesicles (EVs) to participate in BC progression. This study demonstrated that SNHG16 expression was significantly increased in BC tissues and cells. Overexpression of SNHG16 promoted the migration, invasion, and epithelial–mesenchymal transition (EMT) of BC cells. SNHG16 was carried by EVs. Bioinformatics analysis predicted that SNHG16 regulated PPAPDC1A expression by sponging miR-892b, which was confirmed by RNA-fluorescence *in situ* hybridization (FISH), RT-qPCR, dual-luciferase gene reporter assay, and RNA immunoprecipitation (RIP). MDA-MB-157 and HS578T cells were transfected with pcDNA3.1-SNHG16, miR-892b-mimic, or si-PPAPDC1A for functional rescue experiments *in vitro*, and the cells were treated with MDA-MB-231 cell-derived EVs. The results confirmed that enhanced miR-892b expression partially eliminated the increase of migration, invasion, and EMT of BC cells mediated by SNHG16 or EVs. The lung metastasis model in nude mice was established by injecting HS578T cells *via* tail vein. The results showed that si-SNHG16 reduced the metastatic nodules and decreased the vimentin expression. In conclusion, EVs derived from BC cells transferred SNHG16 *via* the miR-892b/PPAPDC1A axis, thus promoting EMT, migration, and invasion of BC.

## Introduction

As the most commonly diagnosed malignancy in women (Libson and Lippman, 2014), breast cancer (BC) initiation is attributed to multiple risk factors, such as DNA damage and genetic alteration (Akram et al., 2017). The current therapeutic strategies available for BC patients include hormone therapy, radiotherapy, surgery, and chemotherapy (Akram et al., 2017). Still, the prognosis of patients with recurrent or metastatic BC is poor, and treatment options must strike a balance between prolonging life and reducing treatment pain (Maughan et al., 2010). Particularly, the vast majority of BC deaths are not because of the primary tumor itself, but due to tumor metastasis to other organs, and consequently, there is an urgent need to control BC recurrence or metastasis (Kozlowski et al., 2015).

Extracellular vesicles (EVs) are cell-derived microparticles that exist in body fluids, including microbubbles, exosomes, and apoptotic bodies (Sun et al., 2018). BC cell-derived EVs are reported to facilitate cancer cell proliferation and oncogene amplification (Keklikoglou et al., 2019). Additionally, EVs also promote the processes conducive to cancer progression, such as extracellular matrix remodeling, angiogenesis induction, and pre-metastasis niche initiation (Wang and Gires, 2019; Kalluri, 2016). For example, EVs derived from aggressive subclones of the triple-negative BC cells tend to transfer the aggressive phenotype to a group of BC cell lines and transmit angiogenesis signal to endothelial cells (O’Brien et al., 2013). Nevertheless, the potential participation of EVs in the progression of BC metastasis is poorly understood.

Mechanically, tumor cell-derived EVs can interact with immune cells, endothelial cells, and tumor-associated fibroblasts in tumor microenvironment by transferring RNA, proteins, lipids, and nucleic acids, thus promoting tumor progression (Deepak et al., 2020). Long non-coding RNAs (lncRNAs) are a class of non-coding RNA transcripts with more than 200 nucleotides, taking part in the tumor initiation and progression widely (Cheng et al., 2018). Aberrant expression of lncRNAs can be observed in BC patients, and the potential clinical applications of lncRNAs in BC have also been unveiled (Niknafs et al., 2016). LncRNA SNHG16 is commonly accepted as an oncogene implicated in the progression of human cancers (Liao et al., 2019). Accumulating studies have revealed that SNHG16 is associated with poor prognosis and metastasis of a variety of human cancers, including BC (Yang and Wei, 2019; Xiao et al., 2020). BC cell-derived exosomes can transfer SNHG16 to γδT1 cells, and CD73 + γδT1 cells are the main regulatory T cells in BC, which play an immunomodulatory role in tumor microenvironment (Salmena et al., 2011; Ni et al., 2020) have proposed a competing endogenous RNA (ceRNA) mechanism in which lncRNA, microRNA (miRNA), and mRNA can achieve crosstalk among each other through forming a regulatory network. The ceRNA network may play a vital role in the progression and metastasis of various cancers, such as colorectal cancer, pancreatic cancer, and liver cancer (Zhong et al., 2019). Intriguingly, Cai et al. (2017) have suggested that SNHG16 induces BC cell migration by competitively binding miR-98. Du (2020) has also shown that the SNHG16/miR-30a axis facilitates BC cell proliferation and invasion by modulating RRM2 expression. However, whether BC cell-EVs mediate SNHG16-related ceRNA communication to promote BC metastasis remains to be determined. This study investigated the role of EVs in BC metastasis by carrying lncRNA SNHG16, along with its ceRNA mechanism, which shall shed light on the management of metastatic BC.

## Materials and Methods

### Ethics Statement

This study got the permission of the Ethical Committee of Tongji Hospital on animal experiment. All the animal experiments were implemented on the guide for the care and use of laboratory animals.

### Bioinformatics Analysis

MicroRNA microarray dataset GSE26659 in BC (containing 77 cancer samples and 17 normal samples) and mRNA dataset GSE61304 (containing 58 cancer samples and four normal samples) were obtained from GEO database^1^. With the normal samples acting as the control, the microarray were differentially analyzed using the limma package in R language and the difference *p*-value was adjusted by false discovery rate (FDR). Differentially expressed genes in BC were screened with the criteria of | logFC| > 2 and FDR < 0.05. The differential expressions of lncRNAs and mRNAs in BC samples and normal samples collected by TCGA and GTEx were searched through GEPIA2 database^2^. The downstream miRNAs of SNHG16 were predicted through RNA22 database^3^, and the target binding sites of lncRNA-miRNA were obtained. The target genes of miR-892b were predicted through TargetScan database^4^, and the binding sites of miRNA-mRNA were obtained. The survival analysis of lncRNA SNHG16, miR-1298-5p, and PPAPDC1A in BC patients was performed through pancancer analysis platform ENCORI^5^ and UALCAN cancer database^6^. The correlation of miR-892b expression with SNHG16 and PPAPDC1A in BC patients was predicted through pancancer co-expression analysis platform ENCORI^7^.

### Dual-Luciferase Gene Reporter Assay

The binding sites of lncRNA SNHG16 and miR-892b, and miR-892b and PPAPDC1A were predicted through RNA22 database (see text footnote 3) and TargetScan database^8^. The complementary binding sequence and mutant sequence of miR-892b with lncRNA SNHG16 and PPAPDC1A were amplified and cloned into pGL4.17 dual-luciferase gene reporter vector (Promega, Madison, WI, United States). The mutant-type plasmids (pGL4.17-SNHG16-MUT and pGL4.17-PPAPDC1A-MUT) and wild-type plasmids (pGL4.17-SNHG16-WT and pGL4.17-PPAPDC1A-WT) were constructed and then transfected with mimic NC or miR-892b mimic (GenePharma, Shanghai, China) into HEK293T cells (Procell Life Science and Technology Co., Ltd., Wuhan, Hubei, China). The luciferase activity was detected 48 h later.

### RNA Immunoprecipitation

RNA immunoprecipitation (RIP) assay was performed in line with the instructions of EZ-Magana RIP kit (17-701, Millipore, Billerica, MA, United States). The cells were lyzed with protease inhibitor and RIP lysis buffer. The magnetic beads were coupled with anti-Ago2 (1:30, ab186733, Abcam Inc., Cambridge, MA, United States) antibody or IgG antibody (ab172730, Abcam), and then cell lysis buffer was added for 6 h incubation at 4°C. The samples were treated with proteinase K solution, and the RNA was extracted by TRIzol method. After removing the beads, the RNA was purified and detected using reverse transcription quantitative polymerase chain reaction (RT-qPCR).

### Cell Culture and Treatment

MDA-MB-231 cells were purchased from the Shanghai Institute of Cellular Biology of Chinese Academy of Sciences, Shanghai, China (Shanghai, China). ZR-75-30 cells were purchased from JRDUN Biotechnology Co., Ltd. (Shanghai, China). HS578T, MCF-10A, and BT474 cells were purchased from LYD Biotechnology Co., Ltd. (Beijing China). MDA-MB-157 cells were purchased from Yuchi Biotechnology Co., Ltd. (Shanghai, China). MDA-MB-231, ZR-75-30, and HS578T cells were cultured in Dulbecco’s modified Eagle’s medium (DMEM; Gersion Biotechnology, Beijing, China) containing 10% fetal bovine serum (FBS; Applygen, Beijing China) and 1% penicillin-streptomycin (WISENT, Nanjing, Jiangsu, China). BT474 cells were cultured in MEM (Sigma-Aldrich, Merck KGaA, Darmstadt, Germany). MCF-10A cells were cultured in RPMI-1640 medium (Sigma-Aldrich) containing 20% FBS, and MDA-MB-157 cells were cultured in Leibovitz’s L-15 medium (Sigma-Aldrich) containing 10% FBS. All the cells were incubated at 37°C with 5% CO_2_. When the cells reached 40–50% confluence, the supernatant was removed and the cells were washed twice with phosphate-buffered saline (PBS). The donor cells were prepared into 2 × 10^6^ cells/mL in 10% FBS medium free of EVs, and incubated for 48 h. Then, the supernatant (Supernate) was collected for subsequent analyses. In some experiments, the cells were treated with 2% FBS containing 10 μM GW4869 (MedChemExpress, Monmouth Junction, NJ, United States) or dimethyl sulfoxide at 37°C for 2 h before collecting the supernatant (Zhou et al., 2017).

### Cell Transfection

miR-892b-mimic, mimic-NC (negative control), si-SNHG16-1, si-SNHG16-2, and si-NC were synthesized by GenePharma Co., Ltd. (Shanghai, China). pcDNA3.1 and pcDNA3.1-SNHG16 were synthesized by Hanbio Biotechnology Co., Ltd. (Shanghai, China). The cell transfection was conducted using Lipofectamine 3000 (Invitrogen Inc., Carlsbad, CA, United States) and HiPerFect transfection reagent (Qiagen GmbH, Hilden, Germany).

### Extraction and Treatment of EVs

The cell supernatant was centrifuged at 500 *g* × 10 min and 2,000 *g* × 20 min to remove the floating cells and cell debris, and then centrifuged at 20,000 *g* × 30 min at 4°C to remove the precipitate and collect the supernatant. After centrifugation at 100,000 *g* × 70 min, the precipitate was the EVs (Wang et al., 2018). The EVs precipitate was washed with PBS, centrifuged again at 100,000 *g* × 70 min, and suspended in 1 mL PBS. The suspension was placed on the top of 30% sucrose cushions to form a clear interface layer, and centrifuged at 100,000 *g* × 70 min at 4°C. The PBS layer was discarded, and the deuteroxide layer was retained. The deuteroxide was mixed with at least five times the volume of PBS, and centrifuged again at 100,000 *g* × 70 min to obtain the purified EVs. The EVs were filtered and sterilized with 0.22 μm membrane, and then put into aseptic Ependorf tube. The EVs were grouped and frozen at −80°C. The EVs of some groups were incubated with 1 μg/mL ribonuclease A (Sigma-Aldrich) at 37°C for 30 min or treated with 0.1% Triton × 100 (Beyotime, Shanghai, China) for 30 min (Wang et al., 2018) for subsequent analysis.

### Identification and Quantification of EVs

The expressions of positive markers (CD9 and CD81) and negative marker (GRP94) of EVs were detected using Western blotting. Bicinchoninic acid (BCA) assay kit (Sigma-Aldrich) was used to quantify the EVs (Zhang R. et al., 2017). The structure and morphology of EVs were observed under transmission electron microscopy (TEM). The extracted EVs were resuspended in PBS, dripped into 100-mesh copper grid, stained negatively with 2% phosphotungstic acid, dried for 15–20 min, and observed under 80 kV TEM (FEI Tecnai G2 Spirit, Thermo Fisher Scientific Inc., Waltham, MA, United States) (Liu et al., 2020). The EVs after PBS dilution were observed by Nanosight NS300 (Malvern, Worcestershire, United Kingdom). The size and concentration of EVs were tracked and measured according to the Brownian motion and diffusion coefficient, with the filtered PBS as the control. Each sample was measured three times (Zhang R. et al., 2017).

### PKH26 Fluorescent Labeling

Extracellular vesicles were labeled using PKH26 Red Fluorescent Cell Linker kit (Sigma-Aldrich). The EVs–dye complex was added with PBS, and centrifuged at 120,000 *g* × 70 min to remove the unbound PKH26. The labeled EVs were incubated with receptor cells on eight-well chamber slides for 3 h. The receptor cells were fixed with 4% paraformaldehyde (Energy Chemical, Shanghai, China) and permeated with 0.1% Triton X-100 (Sigma-Aldrich) and stained with 4′,6-diamidino-2-phenylindole (DAPI; BBI, Shanghai, China) for 30 min. After PBS washing, the cells were observed under Leica DMIRE2 confocal microscope.

### Transwell Assays

Breast cancer cells were resuspended in serum-free medium, and 2 × 10^5^ cells were seeded into 8.0 μm Transwell chamber (Corning Glass Works, Corning, NY, United States), with the basolateral chamber containing serum medium. After 24 h, the Transwell chamber was taken out, and the cells were fixed with methanol and stained with 0.5% crystal violet for 15 min. The non-migrated cells in the apical chamber were gently wiped off with a cotton swab. Following washing with PBS for three times, the migrated cells were photographed and counted. Matrigel (Corning) was added into the apical chamber in advance to detect the invasion ability of cells, and the other steps were the same as before.

### Immunofluorescence Staining

The cells were fixed 4% paraformaldehyde, permeated with 0.2% Triton X-100 (Sigma-Aldrich), and blocked with 5% bovine serum albumin (BSA) (Gersion Biotechnology). The cells were incubated with the primary antibodies E-cadherin (1:200, 60335-1-Ig) and N-cadherin (1:200, 66219-1-Ig) (both purchased from Proteintech, Rosemont, IL, United States) at 4°C overnight, and then with the secondary antibody Alexa Flour 488 labeled goat anti-mouse IgG (D110090-0100, 1:200, BBI). DNA was stained with DAPI (Abcam). The fluorescent microscopy (Leica DMi8) was used for imaging analysis, and the samples only incubated with the secondary antibody were used as the negative control (Blank).

### Fluorescence *in situ* Hybridization

Specific SNHG16 probe and labeled probe (label yellow fluorescence) were designed and synthesized by Nuowo Antai Biotechnology (Beijing, China); RNA visualization *in situ* hybridization reagent (protease, lotion, DAPI, etc.) was purchased from Nuowo Antai Biotechnology. The cells were seeded on the cover glasses, fixed in 4% paraformaldehyde for 20 min, washed with PBS, and incubated overnight in 70% ethanol at 4°C. The next day, the cells were incubated in the washing solution (10% formamide + 2 × SSC) for 5 min. Then, the cover glass was transferred face down to 100 μL hybridization buffer (10% formamide + 2 × SSC + 10% dextran sulfate) containing 125 nM probe, and incubated in a humidification chamber covered with sealing membranes in the dark at 37°C overnight. After hybridizing, the cover glasses were washed with a new washing solution twice (30 min/time) and then washed with 1 × PBS for a short time. DNA was counterstained with DAPI, and the cells were washed with PBS twice. Leica DMIRE2 confocal microscope was used for imaging observation.

### Lung Metastasis Model in Nude Mice

HS578T cells were used for the establishment of lung metastasis model. Totally 24 female nude mice (aged 4–6 weeks) were purchased from Vital River Laboratory Animal Technology Co., Ltd. (Beijing, China) [SYXK (Beijing) 2016-0011]. The nude mice were kept in specific pathogen-free animal room for about 1 week. HS578T cells in logarithmic phase were detached with trypsin and resuspended, washed twice with PBS, and centrifuged at 500 *g* × 5 min, and then the supernatant was discarded. Then, 2 × 10^6^ cells were resuspended in 150 μL PBS and injected into mice *via* tail vein. One day later, the nude mice were allocated into different treatment groups with six mice in each group. MDA-MB-231 cell-derived EVs (100 μg/100 μL) or the same volume of the cell supernatant was injected into mice *via* tail vein twice a week. After 4 weeks, all the mice were sacrificed. The number of metastatic nodules in lungs was counted, and immunohistochemical staining was performed.

### Hematoxylin and Eosin Staining

The cut lung tissues were fixed in 10% paraformaldehyde overnight, washed twice with PBS, dehydrated with gradient ethanol, cleared with xylene solution, embedded in paraffin, sliced into 5 μm sections, and then extended in distilled water at 42°C. The slides were baked in the incubator at 65°C, treated with xylene and gradient ethanol, then stained with hematoxylin and eosin (HE) staining kit (Solarbio, Beijing, China), dehydrated with ethanol again, cleared with xylene, sealed with neutral gum, and observed under microscope.

### Immunohistochemistry

The protein level of vimentin (ab27608, Abcam) in formalin-fixed and paraffin-embedded tissues was detected using immunohistochemistry. Formalin-fixed and paraffin-embedded tissue sections were dewaxed in xylene, rehydrated with graded ethanol, and then boiled in 10 mm citric acid buffer (pH 6.0) for 30 min for antigen repair. The sections were treated with 3% hydrogen peroxide for 10 min to inhibit the activity of endogenous peroxidase. The slides were sealed with 5% BSA (Gersion Bio-technology, Beijing, China), incubated with diluted primary antibody at 4°C overnight, and then incubated with the secondary antibody (ab96899, Abcam) at 37°C for 1 h. The slides were developed with 2,4-diaminobutyric acid (DAB), counterstained with hematoxylin, and examined under the microscope. The percentage of positive cells in tumor tissues was scored respectively: 0, <5%; 1, 5% ∼<25%; 2, 25% ∼<50%; 3, 50% ∼<75%; 4, >75%.

### RT-qPCR

Total RNA was extracted from EVs using SeraMir (System Biosciences, Mountain View, CA, United States), and total RNA was extracted from cells using TRIzol reagent (Invitrogen). The concentration and purity of RNA were determined by UV spectrophotometer. Then, 1 μg total RNA was reverse transcribed into cDNA using High Capacity cDNA reverse transcription kit (Applied Biosystems, Inc., Carlsbad, CA, United States). RT-qPCR was performed using Fast Start Universal SYBR Green Master (Roche Applied Science, Mannheim GmbH, Penzberg, Germany). Relative expression of genes was examined by 2^–Δ^ ^Δ^ ^*Ct*^ method, with GAPDH or U6 as the internal reference. The primer sequence was synthesized by GenePharma (Table 1).

**TABLE 1:** Primer sequence for RT-qPCR.

Gene	Forward (5′–3′)	Reverse (5′–3′)
LncRNA SNHG16	GCAGAATGCCATGGTTTCCC	GGACAGCTGGCAAGAGACTT
miR-892b	GGGCACTGGCTCCTTTCTG	CAGTGCGTGTCGTGGAGT
miR-486-5p	GGGTCCTGTACTGAGCTGC	CAGTGCGTGTCGTGGAGT
miR-139-5p	GGGTCTACAGTGCACGTGTC	CAGTGCGTGTCGTGGAGT
PPAPDC1A	CATTGAGATCGGGGTGCGAG	AGGAATCTTGCCAGTGATGCT
U6	CTCGCTTCGGCAGCACA	AACGCTTCACGAATTTGCGT
GAPDH	GATTGTTGCCATCAACGACC	GTGCAGGATGCATTGCTGAC

### Total Protein Extraction

The cells were collected, lyzed in radio-immunoprecipitation assay (RIPA) buffer (Wako, Osaka, Japan), and ultrasonic treated three times (15 s/time). The supernatant was centrifuged at 15,000 *g* × 10 min as the whole cell protein extract. The EVs were lyzed in five times concentration of RIPA buffer, ultrasonically treated for 5 min, incubated on ice for 15 min, and boiled with six times volume of sample buffer (Nacalai tesque, Germany) to use as the EVs protein extract.

### Western Blotting

An equal amount of protein extract was separated on 12% SDS-PAGE and transferred onto polyvinylidene fluoride membranes (Millipore). The membranes were cultured with the primary antibodies at 4°C overnight, and then with the secondary antibody for 2 h. Next, the membranes were developed and visualized using the enhanced chemiluminescence reagent (Millipore). The protein bands were analyzed using Quantity One (Bio-Rad Laboratories, Hercules, CA, United States). The primary antibodies used in this study were as follows: mouse monoclonal antibody N-cadherin (1:2,000, 66219-1-Ig, Proteintech), mouse monoclonal antibody E-cadherin (1:2,000, 60335-1-Ig, Proteintech), mouse monoclonal antibody vimentin (1:10,000, 60330-1-Ig, Proteintech), mouse monoclonal anti-CD9 (1:2,000, 60232-1-Ig, Proteintech), mouse monoclonal anti-CD81 (1:3,000, 66866-1-Ig, Proteintech), mouse monoclonal antibody GRP94 (1:1,000, 60012-1-Ig, Proteintech), rabbit polyclonal antibody PPAPDC1A (1 μg/mL, PA5-20864, Invitrogen), and mouse monoclonal antibody GAPDH (1:20,000, 60004-1-Ig, Proteintech). The secondary antibodies used in this study were horseradish peroxidase (HRP)-labeled goat anti-mouse IgG (1:2,000, bs-0296G-HRP, Bioss, Beijing, China) and HRP-labeled goat anti-rabbit IgG (1:2,000, bs-0295G-HRP, Bioss).

### Statistical Analysis

Data analysis was introduced using the SPSS 21.0 (IBM Corp., Armonk, NY, United States) and GraphPad Prism 6.0 (GraphPad Software Inc., San Diego, CA, United States). Kolmogorov–Smirnov method checked that the data were in normal distribution. Data are expressed as mean ± standard deviation. One-way or two-way analysis of variance (ANOVA) was employed for the comparisons among multiple groups, followed by Tukey’s multiple comparisons test. The *p*-value was obtained from a two-tailed test, and *p* < 0.05 meant a statistical difference and *p* < 0.01 indicated a very significant difference.

## Results

### LncRNA SNHG16 Was Upregulated in BC Cells

SNHG16 is overexpressed in various cancer tissues and cell lines, participating in the occurrence and progression of cancers (Yang and Wei, 2019). To explore the role of SNHG16 in BC, we screened the differential expression of SNHG16 in BC samples and normal samples collected by TCGA and GTEX databases, and found that SNHG16 expression in BC samples was notably promoted (Figure 1A). We further detected SNHG16 expression in BC cells, and showed that SNHG16 expression in BC cell lines was notably higher than those in immortalized breast epithelial cells (Figure 1B, all *p* < 0.05), with MDA-MB-157 showing the highest expression and HS578T cells showing the lowest expression. UALCAN cancer database showed that the Kaplan–Meier curves of the SNHG16 high expression group and SNHG16 low expression group were different, and the prognosis of the SNHG16 high expression group was worse (Figure 1C, *p* < 0.05).

**FIGURE 1:** LncRNA SNHG16 was upregulated in BC samples and cells. **(A)** The differential expression of lncRNA SNHG16 in BC samples and normal samples collected by TCGA and GTEX databases. The abscissa represents the sample type and the ordinate represents the expression of SNHG16; the red box diagram represents the BC samples and the gray box diagram represents the normal samples, *p < 0.05. **(B)** The expression of SNHG16 in BC cell lines and immortalized breast epithelial cell line was detected using RT-qPCR. **(C)** The survival analysis of SNHG16 in BC patients from UALCAN cancer database. Cell experiment was repeated three times. Data were presented as mean ± standard deviation. Data in **B** were analyzed using one-way ANOVA, followed by Tukey’s multiple comparison test, *p < 0.05 vs. MCF-10A group.

### Overexpression of SNHG16 Promoted Migration and Invasion of BC Cells

LncRNA SNHG16 acts as an oncogene to promote the proliferation, migration, and invasion of BC cells, and also relates to drug resistance and poor prognosis (Cai et al., 2017; Dong et al., 2018b; Kong and Qiu, 2018; Li et al., 2019; Du, 2020). To investigate the effect of SNHG16 on BC metastasis, MDA-MB-157 and HS578T cells were transfected with si-SNHG16-1, si-SNHG16-2, si-NC, pcDNA3.1, and pcDNA3.1-SNHG16. SNHG16 expression of cells in each group is shown in Figure 2A. Epithelial–mesenchymal transition (EMT) is a critical process to promote tumor invasion and metastasis. We then detect the levels of EMT-related proteins (E-cadherin, N-cadherin, and vimentin) using Western blotting. The levels of vimentin and N-cadherin in MDA-MB-157 and HS578T cells were increased significantly after SNHG16 overexpression; the level of E-cadherin was increased, and the levels of vimentin and N-cadherin were decreased after SNHG16 silencing (Figure 2B, all *p* < 0.05). Immunofluorescence further confirmed the EMT phenotype changes in the two BC cells caused by the change of SNHG16 expression (Figure 2C). Next, the effects of SNHG16 on the migration and invasion of BC cells were evaluated using Transwell assay. The results revealed that overexpression of SNHG16 notably enhanced the migration and invasion of MDA-MB-157 and HS578T cells, while silencing SNHG16 showed the opposite trend (Figures 2D,E, all *p* < 0.05). In brief, overexpression of SNHG16 promoted metastasis of BC cells.

**FIGURE 2:** Overexpression of SNHG16 promoted migration and invasion of BC cells. MDA-MB-157 and HS578T cells were transfected with si-SNHG16-1, si-SNHG16-2, si-NC, pcDNA3.1, and pcDNA3.1-SNHG16. **(A)** The expression of SNHG16 was detected using RT-qPCR to verify the transfection efficiency. **(B)** The levels of E-cadherin, N-cadherin, and vimentin were detected using Western blotting. **(C)** The levels of E-cadherin and N-cadherin were detected using immunofluorescence (×200). **(D,E)** The migration and invasion abilities of cells were measured to evaluate the effect of different expressions of SNHG16 on the metastatic ability of BC cells. Cell experiment was repeated three times. Data were presented as mean ± standard deviation. Data in **A, D,** and **E** were analyzed using two-way ANOVA, and data in **B** were analyzed using one-way ANOVA, followed by Tukey’s multiple comparison test, *p < 0.05 vs. pcDNA3.1 group, #*p* < 0.05 vs. si-NC group.

### BC Cell-Derived EVs Carried lncRNA SNHG16

Extracellular vesicles promote intercellular communication in tumor microenvironment by transporting different forms of RNA and protein (Jia et al., 2017). We also speculated that BC cells participated in information transmission and function regulation by the secretion of EVs carrying lncRNA SNHG16. We chose MDA-MB-231 cells, which was commonly used in the research of EVs, for the extraction and identification of EVs. MDA-MB-157 and HS578T were used as receptor cells.

After purification of MDA-MB-231 cell-EVs by centrifugation, hemispherical bilayer vesicle-like structure with a diameter of 50–100 nm was observed under TEM (Figure 3A). Western blotting confirmed the presence of CD9 and CD81, and the absence of GRP94 (Figure 3B), with the GW4869-treated cell supernatant as the control. Nanoparticle tracking analysis showed that the diameters of the isolated EVs were mainly distributed at 90 and 120 nm (Figure 3C). RT-qPCR showed that SNHG16 expression in MDA-MB-231 cell-EVs was not different from that in the cell culture supernatant, but notably higher than that in GW4869-treated cell supernatant (Figure 3D, all *p* < 0.05). To verify that SNHG16 was encapsulated in EVs, we co-incubated RNase A with EVs, and found that SNHG16 expression did not change dramatically, but SNHG16 expression was decreased after co-treatment with ribonuclease A and Triton × 100 (Figure 3E, *p* < 0.05). MDA-MB-231 cell-EVs were further incubated with the receptor cells, and the SNHG16 expression in MDA-MB-157 and HS578T cells was notably upregulated (Figure 3F). The confocal microscope showed that the PKH26-labeled EVs could be encapsulated by the receptor cells (Figure 3G). These results confirmed that MDA-MB-231 cell-EVs were rich in SNHG16 and could be transferred to BC cells by endocytosis, thereby upregulating SNHG16 expression.

**FIGURE 3:** BC cell-EVs carried lncRNA SNHG16. **(A)** The ultrastructure of MDA-MB-231 cell-EVs was observed under TEM. **(B)** The EVs markers (CD9, CD81, and GRP94) were detected using Western blotting. **(C)** The diameter distribution of EVs was detected using Nanoparticle tracking analysis. **(D)** The expression of SNHG16 in MDA-MB-231 cell-EVs, supernatant (Supernate), and GW4869-treated supernatant was detected using RT-qPCR. **(E)** The expression of SNHG16 in EVs treated with ribonuclease A or co-treated with Triton × 100 was detected using RT-qPCR. **(F)** The expression of SNHG16 in MDA-MB-157 and HS578T cells co-incubated with MDA-MB-231 cell-EVs was detected using RT-qPCR. **(G)** PKH26-labeled EVs were encapsulated by MDA-MB-157 and HS578T cells. Cell experiment was repeated three times. Data were presented as mean ± standard deviation. Data in **D** and **E** were analyzed using one-way ANOVA, and data in **F** were analyzed using two-way ANOVA, followed by Tukey’s multiple comparison test, *p < 0.05 vs. EVs group, #*p* < 0.05 vs. control group.

### BC Cells-Secreted EVs Promoted Migration and Invasion of BC Cells by Carrying SNHG16

To determine the effect of EVs, we treated MDA-MB-231 cells with GW4869, and then extracted the cell supernatant to co-incubate with MDA-MB-157 and HS578T cells. Compared with EVs-treated cells, the Supernate/GW4869-treated cells showed reduced SNHG16 expression (Figure 4C, all *p* < 0.05), increased E-cadherin, and decreased vimentin and N-cadherin (Figure 4D, all *p* < 0.05), as well as inhibited migration and invasion ability (Figures 4F,G, all *p* < 0.05). We transfected si-SNHG16-1 into MDA-MB-231 cells to clarify whether EVs affected the receptor cells by carrying SNHG16. RT-qPCR results showed that SNHG16 expression in receptor cells and EVs was reduced after transfection (Figures 4A,B, all *p* < 0.05). MDA-MB-157 and HS578T cells were treated with si-SNHG16-1-transfected EVs, and the results demonstrated that the receptor cells showed reduced SNHG16 expression (Figure 4C, all *p* < 0.05), promoted E-cadherin, and decreased vimentin and N-cadherin (Figure 4D, all *p* < 0.05), as well as inhibited migration and invasion abilities (Figures 4F,G, all *p* < 0.05). The results of immunofluorescence were consistent with that of Western blotting (Figure 4E). In brief, BC cell-EVs promoted BC cell migration and invasion by carrying SNHG16.

**FIGURE 4:** BC cell-EVs promoted BC cell migration and invasion by carrying SNHG16. MDA-MB-231 cells were treated with si-SNHG16 or GW4869, and then EVs or supernatant was extracted and incubated with MDA-MB-157 and HS578T cells. **(A)** The expression of SNHG16 in MDA-MB-231 cells after transfection was detected using RT-qPCR, *p < 0.05 vs. control group. **(B)** The expression of SNHG16 in MDA-MB-231 cell-EVs after transfection was detected using RT-qPCR, *p < 0.05 vs. control group. **(C)** The expression of SNHG16 in MDA-MB-157 and HS578T cells after GW4869/Supernatant or EVs treatment was detected using RT-qPCR. **(D)** The levels of E-cadherin, N-cadherin, and vimentin were detected using Western blotting. **(E)** The levels of E-cadherin and N-cadherin were detected using immunofluorescence (×200). **(F,G)** The migration and invasion abilities of MDA-MB-157 and HS578T cells were measured using Transwell assays. Cell experiment was repeated three times. Data were presented as mean ± standard deviation. Data in **A, B,** and **D** were analyzed using one-way ANOVA, and data in **C, F,** and **G** were analyzed using two-way ANOVA, followed by Tukey’s multiple comparison test, *p < 0.05 vs. control group, #*p* < 0.05 vs. EVs/si-NC group.

### LncRNA SNHG16 Sponged miR-892b to Regulate PPAPDC1A

To further elucidate the mechanism of SNHG16 promoting BC cell migration and invasion, we used LncATLAS^9^ to predict the subcellular localization of SNHG16. SNHG16 was mainly located in the cytoplasm (Figure 5A). RNA FISH confirmed that SNHG16 was mainly distributed in the cytoplasm of MDA-MB-157 cells (Figure 5B). We speculated that SNHG16 was bound to miRNA and played a role in regulating gene expression at the post transcriptional level through ceRNA mechanism. BC miRNA microarray was obtained from GEO database, and it showed that 21 miRNAs were notably poorly expressed in BC samples (Figure 5C). Subsequently, we predicted the downstream miRNAs of SNHG16 through RNA22 database, and took the intersection between the predicted results and the significantly downregulated miRNAs in the microarray analysis (Figure 5D). Three miRNAs (miR-139-5p, miR-892b, and miR-486-5p) were in the intersections of the two sets of data. The expressions of the three miRNAs in MDA-MB-157, HS578T, and MCF-10A cells were detected, and miR-892b showed the most differential expression (Figure 5E, all *p* < 0.05). Relatively little was known about the function of miR-892b in BC, so we chose miR-892b as the downstream object of SNHG16 in this study. We predicted the co-expression of SNHG16 and miR-892b in BC patients through ENCORI pancancer analysis database, and the results showed that there was no significant correlation between them (Supplementary Figure 1A, *p* > 0.05), and miR-892b showed extremely poor expression in most tumor samples, so these clinical sample data cannot reflect the regulatory effect between SNHG16 and miR-892b. Moreover, the survival status of miR-892b in BC patients was inquired through ENCORI pancancer analysis database. It was found that there was no difference in Kaplan–Meier curve between miR-892b high expression and low expression groups (Figure 5F). However, Jiang et al. (2016) reported that miR-892b expression was downregulated in human BC samples and was correlated with poor survival, indicating the involvement of miR-892b in the pathogenesis of BC and its research value. miR-892b expression in MDA-MB-157 and HS578T cells was detected. Compared with the control cells, the si-SNHG16-1-transfected cells had elevated miR-892b expression and the pcDNA3.1-SNHG16-transfected cells had reduced miR-892b expression (Figure 5G, all *p* < 0.05). The binding relationship between miR-892b and lncRNA SNHG16 was verified using dual-luciferase gene reporter assay, and the results demonstrated that the luciferase activity of HEK293T cells co-transfected with pcDNA3.1-SNHG16-WT and miR-892b mimic was significantly reduced (Figure 5H, *p* < 0.05), confirming the target binding of miR-892b and lncRNA SNHG16. It is well known that mature miRNAs can form RNA-induced silencing complexes with Ago protein family to degrade target genes or inhibit transcription (Stavast and Erkeland, 2019). Therefore, we used anti-Ago2 antibody to conduct RIP assay in MDA-MB-157 and HS578T cells, and the results showed that SNHG16 and miR-892b could bind to Ago2 at the same time (Figure 5Q).

**FIGURE 5:** LncRNA SNHG16 sponged miR-892b to regulate PPAPDC1A. **(A)** SNHG16 was mainly located in the cytoplasm through LncATLAS prediction. **(B)** RNA FISH confirmed that SNHG16 was distributed in the cytoplasm of MDA-MB-157. **(C)** The heat map of downregulated miRNAs in BC in the GSE26659, the abscissa is the sample number and the ordinate is the miRNA name; the histogram at the top right is the color scale. **(D)** The intersection between the prediction results of RNA22 database for the downstream miRNAs of SNHG16 and the downregulated miRNAs in GSE26659; the two circles in the panel show the prediction results of RNA22 and the results of microarray analysis, and the middle part shows the intersection of the two set of data. **(E)** The expressions of miR-139-5p, miR-892b, and miR-486-5p in MDA-MB-157, HS578T, and MCF-10A cells were detected using RT-qPCR. **(F)** Kaplan–Meier curve of miR-892b in BC patients from ENCORI pancancer database. **(G)** MDA-MB-157 and HS578T cells were transfected with pcDNA3.1-SNHG16 and si-SNHG16, and the expression of miR-892b was detected using RT-qPCR. **(H)** The binding relationship between SNHG16 and miR-892b was verified using dual-luciferase gene reporter assay. **(I)** The heat map of downregulated genes in BC in the GSE61304. **(J)** Intersection of miR-892b target genes predicted by TargetScan and upregulated genes in GSE61304. **(K)** Differential expression of PPAPDC1A in BC samples and normal samples collected by TCGA and GTEx database. **(L)** Kaplan–Meier curve of PPAPDC1A in BC patients from UALCAN pancancer database. **(M)** MDA-MB-157 and HS578T cells were transfected with pcDNA3.1-SNHG16 and si-SNHG16, and the PPAPDC1A mRNA expression was detected using RT-qPCR. **(N)** The binding relationship between PPAPDC1A and miR-892b was verified using dual-luciferase gene reporter assay. **(O)** MDA-MB-157 and HS578T cells were treated with EVs or GW4869/Supernatant, and the expression of miR-892b was detected using RT-qPCR. **(P)** MDA-MB-157 and HS578T cells were treated with EVs or GW4869/Supernatant, and PPAPDC1A mRNA expression was detected using RT-qPCR. **(Q)** Anti-Ago2 RNA immunoprecipitation assay was used to detect the enrichment of SNHG16, miR-892b, and PPAPDC1A mRNA in the immunoprecipitation complex, with IgG as control. Cell experiment was repeated three times. Data were presented as mean ± standard deviation. Data in **E, G, M, O,** and **P** were analyzed using one-way ANOVA, and data in **H** and **N** were analyzed using two-way ANOVA, followed by Tukey’s multiple comparison test, *p < 0.05.

To further explore the downstream mechanism of miR-892b, we predicted the target genes of miR-892b through TargetScan database. Meanwhile, BC mRNA microarray was obtained from GEO database, and it showed that 57 genes were increased in BC (Figure 5I). Four genes were found in the intersections of upregulated genes and target genes (Figure 5J). Among the four genes, PPAPDC1A was upregulated notably in BC (Table 2), and there were few studies about the role of PPAPDC1A in BC. Furthermore, we searched the TCGA and GTEx databases for PPAPDC1A expression in BC (Figure 5K), and found that PPAPDC1A was highly expressed in BC. ENCORI pancancer co-expression analysis predicted that there was no correlation between the expression of miR-892b and PPAPDC1A (PLPP4) in BC patients (Supplementary Figure 1B, *p* > 0.05) and miR-892b showed extremely poor expression in most clinical tumor samples, so these clinical sample data cannot reflect the regulatory effect between PPAPDC1A and miR-892b. According to the UALCAN cancer database, although there was no significant difference in the survival curve of BC patients with different PPAPDC1A expression, the long-term survival rate of patients with high PPAPDC1A expression showed a lower trend (Figure 5L). RT-qPCR demonstrated that PPAPDC1A mRNA expression in si-SNHG16-1-transfected cells was decreased, but was increased in pcDNA3.1-SNHG16-transfected cells (Figure 5M, all *p* < 0.05). Similarly, the binding relationship between miR-892b and PPAPDC1A mRNA was verified using dual-luciferase gene reporter assay and RIP assay (Figures 5N,Q). Based on the above results, we hypothesized that SNHG16 upregulated PPAPDC1A expression by sponging miR-892b, thus playing an oncogenic role in BC.

**TABLE 2:** Differential expression of candidate genes in GSE61304.

Symbol	logFC	*p*-value	Adj *P*-value
PPAPDC1A	2.443459112	1.08E-07	4.24E-05
NUF2	2.276483656	1.25E-07	4.37E-05
RRM2	2.13793638	1.49E-07	4.91E-05
MMP9	2.033663415	1.18E-06	0.000187388

To verify the effect of EVs on the expressions of miR-892b and PPAPDC1A in receptor cells, we measured the expressions of miR-892b and PPAPDC1A in MDA-MB-157 and HS578T cells treated with Supernate/GW4869 or EVs. The results exhibited that EVs-treated cells showed decreased miR-892b expression and increased PPAPDC1A mRNA expression, compared with Supernate/GW4869-treated cells (Figures 5O,P, all *p* < 0.05). To verify whether EVs functioned by carrying SNHG16, we treated receptor cells with EVs/si-NC and EVs/si-SNHG16-1. EVs/si-SNHG16-1-treated cell showed increased miR-892b expression and decreased PPAPDC1A mRNA expression (Figures 5O,P, all *p* < 0.05). Therefore, we further hypothesized that BC cells transferred SNHG16 to receptor cells by secreting EVs, and played a role *via* miR-892b/PPAPDC1A.

### SNHG16 Carried by EVs Promoted Migration and Invasion of BC Cells by Inhibiting miR-892b and Upregulating PPAPDC1A

To verify the regulatory effect of miR-892b on PPAPDC1A, we transfected MDA-MB-157 and HS578T cells with miR-892b mimic and si-PPAPDC1A, followed by the EVs treatment. Compared with EVs + mimic-NC-treated cells, EVs + miR-892b-mimic-treated cells showed increased miR-892b expression and decreased PPAPDC1A mRNA expression; compared with EVs + si-NC-treated cells, EVs + si-PPAPDC1A-treated cells showed reduced miR-892b and PPAPDC1A mRNA expression (Figure 6A, all *p* < 0.05). Western blotting revealed that the protein level of PPAPDC1A in EVs + miR-892b-mimic and EVs + si-PPAPDC1A groups was decreased (Figure 6B, all *p* < 0.05), and the migration and invasion of the two groups were weaker than those of the control group (Figures 6C,D, all *p* < 0.05). To confirm that SNHG16 regulated PPAPDC1A expression by sponging miR-892b, we co-transfected MDA-MB-157 and HS578T cells with pcDNA3.1-SNHG16 and miR-892b-mimic for rescue experiments, with pcDNA3.1 empty vector and mimic NC as control. RT-qPCR and Western blotting results showed that miR-892b-mimic could reverse the increase of PPAPDC1A mRNA expression and protein level induced by pcDNA3.1-SNHG16 (Figures 6E,F, all *p* < 0.05). These results suggested that miR-892b mimic and si-PPAPDC1A attenuated the promoting effect of SNHG16 on the migration and invasion of BC cells *in vitro*, and confirmed that miR-892b/PPAPDC1A axis was involved in the downstream regulation of SNHG16.

**FIGURE 6:** SNHG16 carried by EVs promoted migration and invasion BC cells by inhibiting miR-892b and upregulating PPAPDC1A. MDA-MB-157 and HS578T cells were transfected with miR-892b-mimic or si-PPAPDC1A, followed by MDA-MB-231 cell-EVs treatment. **(A)** The miR-892b and PPAPDC1A expression in MDA-MB-157 and HS578T cells was detected using RT-qPCR. **(B)** The PPAPDC1A protein level in MDA-MB-157 and HS578T cells was detected using Western blotting. **(C,D)** The migration and invasion of MDA-MB-157 and HS578T cells were measured using Transwell assays. MDA-MB-157 cells and HS578T cells were treated with pcDNA3.1-SNHG16 and miR-892b-mimic. **(E)** PPAPDC1A mRNA expression in cells was detected using RT-qPCR. **(F)** PPAPDC1A protein level in cells was detected using Western blotting. Cell experiment was repeated three times. Data were presented as mean ± standard deviation. Data in **A** and **B** were analyzed using one-way ANOVA, and data in **C** and **D** were analyzed using two-way ANOVA, followed by Tukey’s multiple comparison test, *p < 0.05 vs. EVs + mimic-NC group, #*p* < 0.05 vs. EVs + si-NC group; @*p* < 0.05.

### SNHG16 Carried by EVs Promoted Lung Metastasis of BC Cells in Nude Mice

We injected HS578T cells into the mice *via* tail vein to establish the metastasis model. Then, the MDA-MB-231 cell-EVs or GW4869-treated cell supernatant (Supernate/GW4869) was injected into mice. Compared with EVs-treated mice, the Supernate/GW4869-treated mice showed decreased metastatic nodules (Figure 7A, *p* < 0.05). HE staining showed tumor metastatic foci, and immunohistochemical staining confirmed that the expression of vimentin was increased in the EVs group (Figure 7B, *p* < 0.05). These results suggested that EVs promoted the metastasis of BC cells *in vivo*. Then the mice were treated with EVs/si-NC or EVs/si-SNHG16-1. The EVs/si-SNHG16-1-treated mice showed reduced metastatic nodules (Figure 7A, *p* < 0.05) and decreased vimentin expression (Figure 7B, *p* < 0.05). It was suggested that EVs promoted BC metastasis *in vivo* by carrying SNHG16.

**FIGURE 7:** SNHG16 carried by EVs promoted lung metastasis of BC cells in nude mice. HS578T cells were injected into mice *via* tail vein to establish the metastasis model. **(A)** Counting of metastatic lung nodules. **(B)** HE staining and vimentin immunohistochemical staining of metastatic lung tissues, *N* = 6. Data were analyzed using one-way ANOVA, followed by Tukey’s multiple comparison test, ^∗^*p* < 0.05.

## Discussion

The high clinical burdens of metastatic BC highlight the urgent need for better clinical interventions (Kimbung et al., 2015). EVs foster BC progression by facilitating invasion, pre-metastatic niche preparation, evading immune surveillance, and inducing drug resistance (Wang and Gires, 2019). LncRNA SNHG16 can act as a promising therapeutic target in BC (Du, 2020). This study demonstrated that BC-cell EVs promoted BC metastasis by carrying lncRNA SNHG16 *via* the miR-892b/PPAPDC1A axis (Figure 8).

**FIGURE 8:** Mechanism of lncRNA SNHG16 on the miR-892b/PPAPDC1A regulatory axis. The donor BC cell-secreted EVs carried lncRNA SNHG16 into the intercellular matrix, which was then encapsulated by the receptor cells and released SNHG16. The EVs carried SNHG16 competitively bound to miR-892b to inhibit the binding of miR-892b with PPAPDC1A, thus upregulating the expression of PPAPDC1A, promoting epithelial–mesenchymal transition, and ultimately promoting the invasion and metastasis of BC cells.

The upregulation of SNHG16 in cancer cells indicates that SNHG16 may serve as a promising biomarker and therapeutic target for human malignancies (Yang and Wei, 2019). To determine the function of SNHG16 in BC, we screened the differential expression of SNHG16 in BC and normal samples collected by databases, and showed that SNHG16 expression in BC samples was notably promoted. SNHG16 expression in BC cell lines was also notably higher than those in immortalized breast epithelial cells. Consistently, Cai et al. (2017) have demonstrated that SNHG16 expression is frequently upregulated in BC tissues, and SNHG16 may function as an oncogene of BC cell migration. Taken together, lncRNA SNHG16 was upregulated in BC cells. SNHG16 plays a vital role in various hallmarks that determine human cancer, including facilitating proliferation, inducing migration and invasion, as well as affecting chemoresistance (Yang and Wei, 2019). Importantly, EMT has been recognized to trigger cancer invasion and metastasis (Lamouille et al., 2014; Cao et al., 2015). To investigate the effect of SNHG16 on BC metastasis, MDA-MB-157 and HS578T cells were transfected with si-SNHG16-1, si-SNHG16-2, si-NC, pcDNA3.1, and pcDNA3.1-SNHG16. EMT is accompanied by the reduction of epithelial markers (E-cadherin) and the enhancement of mesenchymal markers (*N*-cadherin and vimentin) (Liu et al., 2015). We revealed that the level of E-cadherin was increased, and the levels of vimentin and N-cadherin were decreased in MDA-MB-157 and HS578T cells transfected with si-SNHG16. Zhou et al. (2019) have shown that SNHG16 knockdown can repress EMT and invasion of gastric cancer cells. Transwell assays also exhibited that overexpression of SNHG16 notably enhanced the migration and invasion of MDA-MB-157 and HS578T cells, while downregulation of SNHG16 showed the opposite trend. In brief, overexpression of SNHG16 promoted migration and invasion of BC cells.

Cancer cells-released EVs can regulate the biological characteristics of distant organ niches, thus promoting the growth of metastatic cancer cells (Keklikoglou et al., 2019). BC cells-derived EVs act as a carcinogenic signal, which reprogram systemic energy metabolism and cause cancer-associated cachexia in BC (Wu et al., 2019). EVs occupy a crucial part in intercellular communication in tumor microenvironment *via* transferring lncRNAs (Yang J. et al., 2018). For example, EVs-mediated transfer of lncRNA SNHG14 enhances trastuzumab chemoresistance in BC (Dong et al., 2018a). We also speculated that BC cells participated in information transmission and function regulation by the secretion of EVs carrying lncRNA SNHG16. We isolated MDA-MB-231 cell-EVs and found that MDA-MB-231 cell-EVs were rich in SNHG16 and SNHG16 could be transferred to BC cells, thereby upregulating SNHG16 expression.

Extracellular vesicles-delivered nucleic acid and proteins contribute to the occurrence, metastasis, and drug resistance of BC (Yu et al., 2015; Mashouri et al., 2019). To determine the effect of EVs, we treated MDA-MB-231 cells with GW4869 (EVs inhibitor) and then extracted the cell supernatant to co-culture with MDA-MB-157 and HS578T cells. Compared with EVs-treated cells, the Supernate/GW4869-treated cells showed reduced SNHG16 expression, increased E-cadherin, and decreased vimentin and N-cadherin, as well as inhibited migration and invasion. Briefly, EVs inhibitor downregulated SNHG16 expression and suppressed BC cell migration and invasion. Then, into MDA-MB-231 cells were transfected with si-SNHG16-1 to clarify whether EVs affected the receptor cells by carrying SNHG16. EVs/si-SNHG16-1-treated cells showed promoted E-cadherin and decreased vimentin and N-cadherin, as well as inhibited migration and invasion. It was confirmed that BC cell-EVs promoted BC cell migration and invasion by carrying SNHG16.

Subsequently, we further elucidated the mechanism of SNHG16 promoting BC metastasis. Our experimental results confirmed that SNHG16 was mainly distributed in the cytoplasm of MDA-MB-157 cells. Hence, we speculated that SNHG16 played a role in BC through ceRNA mechanism. The downstream miRNAs of SNHG16 were predicted through RNA22 database, and the intersection between the predicted results and the significantly downregulated miRNAs in the microarray was taken. miR-892b was selected as the downstream research object of SNHG16 in this study. miR-892b is downregulated in BC tissues, which is associated with a low survival rate, and elevated miR-892b expression notably represses cancer growth, metastasis, and angiogenesis (Jiang et al., 2016). Our results exhibited that the si-SNHG16-1-transfected cells had elevated miR-892b expression and the pcDNA3.1-SNHG16-transfected cells had reduced miR-892b expression. We then predicted the target genes of miR-892b through TargetScan database, and found that PPAPDC1A expression was upregulated notably in BC. The involvement of PPAPDC1A in the malignant progression of human cancers has been unveiled (Zhang X. et al., 2017). Particularly, PPAPDC1A is demonstrated to be elevated in estrogen receptor-negative BC patients (Manzano et al., 2014). We showed that PPAPDC1A expression in si-SNHG16-1-transfected cells was decreased, but was increased in pcDNA3.1-SNHG16-transfected cells. To verify the effect of EVs on the expressions of miR-892b and PPAPDC1A, we measured the expressions of miR-892b and PPAPDC1A in MDA-MB-157 and HS578T cells treated with GW4869 cell supernatant or EVs. The results exhibited that EVs-treated cells showed decreased miR-892b expression and increased PPAPDC1A expression. Additionally, EVs/si-SNHG16-1-treated cells showed increased miR-892b expression and decreased PPAPDC1A expression. Briefly, BC cell-EVs transferred SNHG16 to receptor cells and promoted BC metastasis *via* miR-892b/PPAPDC1A. Moreover, functional rescue experiments confirmed that miR-892b mimic and si-PPAPDC1A attenuated the promoting effect of SNHG16 on BC metastasis *in vitro*, and miR-892b/PPAPDC1A axis was involved in the downstream regulation of SNHG16. Tumor xenograft in nude mice also suggested that EVs promoted BC metastasis *in vivo* by carrying SNHG16.

To sum up, we highlighted that BC-cell EVs promoted BC metastasis *via* the lncRNA SNHG16/miR-892b/PPAPDC1A axis based on bioinformatics prediction and functional experiments. This study was the first to demonstrate that EVs promoted intercellular communication of BC by transferring lncRNA SNHG16, thus affecting BC metastasis. There are also some limitations in this study. First, this study focused on the role of EVs in the communication between BC cells, but failed to explore the effects of EVs on tumor-associated fibroblasts, endothelial cells, and tumor microenvironment. Second, the selected BC cell lines in this study were limited, and other commonly used cell lines or clinical specimens of BC should be extended to increase the reliability. Third, EVs are rich in a large number of disease-related RNA molecules, but the choice of internal reference in the detection of exosome RNA is controversial. Notably, most of the tumor samples showed extremely low expression of miR-892b and ENCORI pancancer co-expression analysis predicted that there was no significant correlation between the expression of SNHG16 and miR-892b, and between PPAPDC1A and miR-892b in BC patients. Hence, the data cannot support the existence of the SNHG16-miR-892b-PPAPDC1A circuit in clinical samples. The circuit we observed might be limited in cultured cells and cannot recapitulate in patients. At present, the internal reference used in the detection of exosome RNA is basically PCR internal reference in classical cell biology research, such as GAPDH, β-actin, and 18S, but the use of single internal reference has the following limitations: the accuracy is poor when the RNA expression to be measured is far from the internal reference gene expression; the expression of non-EVs specific internal reference gene may be affected by the extraction method of EVs. Therefore, there is no unified internal reference for exosome RNA of all sample types, and researchers should choose reasonable internal reference according to their own sample types and EVs extraction methods. PCR correction of exoRNA using multiple internal reference genes with different expression abundances is also an option. According to the research of Han et al. (2020), this study selected GAPDH as the internal reference of PCR for exoRNA, because we have similarities in sample types and EVs extraction methods. We will try to use a variety of internal reference genes for PCR correction of exoRNA in the subsequent study.

In future research, we shall further explore the effect of lncRNA SNHG16 carrying EVs on tumor microenvironment, which is a key factor affecting tumor growth and metastasis. Tumor cell-derived EVs participate in the regulation of tumor microenvironment in a variety of ways. EVs shuttle between cells to realize material transport and information exchange by carrying functional proteins, RNA, DNA, and other bioactive substances (Milane et al., 2015). For example, tumor cell-derived EVs can be transferred to vascular endothelial cells, thereby promoting tumor angiogenesis (Maji et al., 2017). Tumor cell-derived EVs induce mesenchymal stem cells to differentiate into tumor-associated fibroblasts (Baroni et al., 2016), and act on immune cells to regulate cytokine expression and promote tumor immune escape (Yang Y. et al., 2018). The current study found that EVs can transmit information among the subpopulations of BC cells. We will explore the effects of EVs on the physiological functions of endothelial cells and tumor-associated fibroblasts and further discover the mechanism of EVs in regulating the tumor environment and promoting the BC progression.

## Data Availability Statement

The original contributions presented in the study are included in the article/Supplementary Material; further inquiries can be directed to the corresponding author/s.

## Ethics Statement

The animal study was reviewed and approved by the Ethical Committee of Tongji Hospital.

## Author Contributions

WX and YL: conceptualization. WX, TC, TX, and MD: validation, research, resources, data reviewing, and writing. WX and XH: review and editing. All authors read and approved the final manuscript.

## Conflict of Interest

The authors declare that the research was conducted in the absence of any commercial or financial relationships that could be construed as a potential conflict of interest.

## Footnotes

1 https://www.ncbi.nlm.nih.gov/geo/

2 http://gepia2.cancer-pku.cn/#index

3 https://cm.jefferson.edu/rna22/

4 http://www.targetscan.org/vert_71/

5 http://starbase.sysu.edu.cn/panGeneSurvivalExp.php

6 http://ualcan.path.uab.edu/analysis.html

7 http://starbase.sysu.edu.cn/panMirCoExp.php

8 http://www.targetscan.org/vert_71/

9 http://lncatlas.crg.eu/

## Supplementary Material

Supplementary Figure 1 Prediction of the co-expression of miR-892b with SNHG16 or PPAPDC1A. **(A)** ENCORI pancancer database was used to predict the correlation between miR-892b and SNHG16 expression in BC patients. **(B)** ENCORI pancancer database was used to predict the correlation between miR-892b and PPAPDC1A (PLPP4) expression in BC patients.
